# Breaching Subjects' Thoughts Privacy: A Study with Visual Stimuli and Brain-Computer Interfaces

**DOI:** 10.1155/2021/5517637

**Published:** 2021-08-09

**Authors:** Mario Quiles Pérez, Enrique Tomás Martínez Beltrán, Sergio López Bernal, Alberto Huertas Celdrán, Gregorio Martínez Pérez

**Affiliations:** ^1^Departamento de Ingeniería de la Información y las Comunicaciones, University of Murcia, Murcia 30100, Spain; ^2^Communication Systems Group (CSG), Department of Informatics (IfI), University of Zürich UZH, CH-8050 Zürich, Switzerland

## Abstract

Brain-computer interfaces (BCIs) started being used in clinical scenarios, reaching nowadays new fields such as entertainment or learning. Using BCIs, neuronal activity can be monitored for various purposes, with the study of the central nervous system response to certain stimuli being one of them, being the case of evoked potentials. However, due to the sensitivity of these data, the transmissions must be protected, with blockchain being an interesting approach to ensure the integrity of the data. This work focuses on the visual sense, and its relationship with the P300 evoked potential, where several open challenges related to the privacy of subjects' information and thoughts appear when using BCI. The first and most important challenge is whether it would be possible to extract sensitive information from evoked potentials. This aspect becomes even more challenging and dangerous if the stimuli are generated when the subject is not aware or conscious that they have occurred. There is an important gap in this regard in the literature, with only one work existing dealing with subliminal stimuli and BCI and having an unclear methodology and experiment setup. As a contribution of this paper, a series of experiments, five in total, have been created to study the impact of visual stimuli on the brain tangibly. These experiments have been applied to a heterogeneous group of ten subjects. The experiments show familiar visual stimuli and gradually reduce the sampling time of known images, from supraliminal to subliminal. The study showed that supraliminal visual stimuli produced P300 potentials about 50% of the time on average across all subjects. Reducing the sample time between images degraded the attack, while the impact of subliminal stimuli was not confirmed. Additionally, younger subjects generally presented a shorter response latency. This work corroborates that subjects' sensitive data can be extracted using visual stimuli and P300.

## 1. Introduction

Technology is closely linked to our daily lives, making it impossible to think about performing some tasks without direct or indirect help. This is mainly due to the constant evolution of technology and the current trend to make it more user-friendly. Consequently, new technologies based on computer-human interaction, such as Kinect devices [1] or Brain-computer interfaces (BCIs), have gained relevance for the last decades. BCIs provide a bidirectional channel between the brain and external devices, enabling two modes of use [2]. On the one hand, BCI can stimulate or inhibit neuronal activity to treat neurodegenerative diseases. On the other hand, they can also monitor brain activity to diagnose diseases or control external devices.

BCIs can be mainly classified into two categories depending on their invasiveness level in the human body [3]. On the one hand, there are invasive interfaces, for which a surgical operation is necessary. This is the case of brain implants [4], which can either pass through the cerebral cortex to measure the activity of single neurons or be implanted on the cerebral cortex surface to measure the activity of groups of neurons. The application scenarios for this type of interface are usually clinical due to the impact on the subjects' physical integrity. On the other hand, noninvasive BCIs have electrodes placed on the head surface to capture the transmission of electrical impulses during brain activity, known as electroencephalography (EEG). In this case, the obtained signal is the aggregation of the neurons located in the area close to the electrodes. In summary, noninvasive BCIs provide less accurate measurements than invasive, as the skull weakens the signal and adds noise. However, the advantage of avoiding the surgery in noninvasive approaches and the price justify why noninvasive BCIs are much more extended than invasive in entertainment scenarios.

Thanks to the evolution of technology associated with BCIs, they have gone beyond the medical field and have reached other sectors such as entertainment and video games [5], where the purpose is to give players a greater sense of immersion. In the same way, the clinical sector has also advanced and expanded the use of these interfaces. For example, the literature has proposed gamification processes, which seek to know the subject's emotional state, subjecting it to a training process called *mindfulness* [6]. Another field of application, where BCI has been tested, is in industrial robotics, where the control of robots is sought to implement significant precision tasks with brain activity [7]. This last application is one of the most promising due to the increment of life expectancy in society. It is associated with a progressive increase in the number of people in a situation of dependence. The evolution towards aging societies demands new solutions to assist the elderly, requiring help to carry out daily life activities. In this sense, BCI systems can be extremely beneficial, as they facilitate a new way of interacting with the different devices existing in their environments [8]. Therefore, BCIs contribute to an increase in the dependent people's autonomy, improving their quality of life and their integration into society.

One of the most well-known application scenarios of BCI is the study of bioelectric potentials produced as a response of the central nervous system to certain stimuli. This is known as “evoked potential” (ERP) [9]. There are several types of evoked potentials, such as visual, auditory, or sensory. Thanks to the study of these evoked potentials, diverse information can be obtained from the subject. For example, the subject's intelligence has been related to the latency of appearance of the evoked potential; the higher the intelligence quotient, the shorter the latency time of the evoked potential [10]. The evoked potential P300 [11] is a response of the brain that occurs about 300 ms after a “significant” event has taken place (hence the name P300, “*P*” since it is a positive increase in brain voltage and “300” because, as mentioned above, it occurs about 300 ms after the event). This potential is mainly observed in the occipital and parietal areas of the cerebral cortex. The events that provoke this wave can be visual and auditory. However, this work focuses on visual stimuli. This potential can be intentionally provoked by following the Oddball paradigm (among others), which is based on randomly showing a series of known stimuli in a set of unknown stimuli. One of the most famous scenarios, where this paradigm has been tested, is with the *P300 Speller*, which, in a very abbreviated form, is a matrix of letters illuminated by rows and columns, whose purpose is to try to guess the character on which the user has placed his attention [12].

In particular, the P300 [11] potential appears when the subject already knew the stimulus presented to him/her. Therefore, malicious use can cause some privacy implications that must be taken into account when using BCIs. The first and most important is to study whether it is possible to obtain sensitive information from the subject through evoked potentials. For example, images can obtain private personal information, such as ideology or sexual orientation. This could apply to people with high relevance, such as the Prime Minister, whose data would be highly valued. On the other hand, if less prominent users are targeted, the attacks could obtain banking information for financial gain. In this sense, Martinovic et al. [13] carried out a series of experiments to obtain bank details or known locations through the P300. The experiment concluded that it was possible to detect when a subject knew a specific visual stimulus. This cybersecurity issue becomes even more dangerous when the stimuli are produced without the subject being aware of them. It is the case of subliminal images or, in other words, images that subjects are not conscious of seeing, but they have been processed by the brain (or not). Moreover, the data obtained and transmitted by BCIs are critical. Because of that, BCI technologies could benefit from the application of existing cybersecurity mechanisms such as blockchain [14], a promising solution to improve the security of the data and prevent attacks affecting the integrity of P300. However, the subliminal aspects of these stimuli are not clear in the literature and are, therefore, an open challenge. Due to the fact that there is only one paper dealing with the impact of subliminal attacks (Frank et al. [15]), many questions remain open about the methodology of these experiments. Some of the issues that are sought to be clarified are as follows: (1) how much time the images should be shown, (2) how much the sampling time of stimuli should be reduced, (3) whether images should be entirely invisible, or (4) whether the reaction is uniform in all subjects, among others. In this context, different parameters should be considered when experimenting in this field. As an example, we highlight the sampling time of the images and the way they appear. Similarly, these images should be shown to a more significant number of subjects, in which different ages and genders should be considered. After this, some new and strong conclusions indicating whether the results are similar to those obtained in the literature experiments should be provided.

To improve some of the previous challenges, the first contribution of this work is the implementation of a BCI framework able to acquire, process, and store the EEG signal to detect a P300 wave. This framework also displays, in a visual way, the EEG signal, which allows detecting if there is a P300 or not. Once the framework is implemented, the second contribution, and the main one, is the creation of a set of experiments, where different videos show known and unknown visual stimuli (following the Oddball paradigm) to different subjects wearing a BCI headset, in which EEG is acquired and managed by the BCI framework to show the P300 wave graphically. The experiments gradually reduce the sampling time of the known stimuli to study how this aspect affects the generation of the P300 wave. They begin with a visible image, shown during 500 ms, and ends with an invisible, or subliminal, image (shown during 10 ms). It is also important to mention that these experiments have been carried out with ten subjects of different ages and gender to obtain the most reliable results. After performing the experiments, it is determined that, for the supraliminal experiments (experiments from one to four), a P300 potential is generated about 50% of the time on average for all subjects. If attention is focused on how characteristics affect the generation of the P300, younger subjects generate P300 potentials with a slightly shorter latency. Concerning the fifth experiment, based on subliminal stimuli, no evidence has been obtained that they generate an impact on the subject's brain.

The remainder of the paper is structured as follows.  Section 2 introduces the related work existing in the literature. After that, Section 3 describes the architecture of the framework built to deal with data acquisition, processing, and visualization developed, followed by an analysis of the experiments and the results obtained. Finally, Section 5 highlights conclusions and future work.

## 2. Related Work

This section reviews the existing literature concerning cybersecurity in BCI, studying possible attacks and emphasizing those focused on attacking the integrity of the user's sensitive information. After that, it analyzes the impact of subliminal stimuli from a psychological perspective, indicating how this issue has been approached over the years and how effective these stimuli are.

### 2.1. Oddball Paradigm and Potential P300

The most common way to induce the generation of a P300 potential has been through the Oddball paradigm [16], based on presenting a known stimulus from a larger set of unknown stimuli [17]. Following this pattern, numerous experiments based on the Oddball paradigm and the generation of P300 potentials have been performed. In these experiments, it is studied how the parameters used to present the stimuli affect the P300 wave [18].

Moving to the application scenarios, in which Oddball and P300 have been used, there are numerous studies proposing many applications for this paradigm (see Figure 1). For example, Campanella et al. [19] performed an experiment, where they combined both visual and auditory stimuli to increase the clinical sensitivity of these P300 modulations like amplitude or latency. Other studies have focused on studying how the different physiological factors of the subject affect the generation of P300, as in Kamp [20], where they focused on the age of the subjects. This paradigm has been extensively used in the medical field, specifically for the detection of mental illnesses such as Parkinson's disease [21], Alzheimer [22], schizophrenia [23], locked-in syndrome [24], or disorders such as anxiety [18].

Thanks to the progress made by BCIs in recent years, these scenarios have been able to go beyond the medical sector and reach other areas. For instance, the video game sector aims to obtain greater immersion while playing [25]. Another area, where they have had a great impact, is robotics. This is based on the control of robots through the P300 potential [7], being useful for people with psychomotor problems, allowing the use of robotic extremities or prostheses. Moreover, Arrichello et al. [26] proposed the creation of an assistant robot to perform manipulation tasks that may help in daily life operations controlled by the P300 potential. Finally, the generation of the potential using the Oddball paradigm has been used for user authentication, for example, based on the recognition of a set of faces [27].

### 2.2. Cybersecurity on BCI

Although BCIs have significantly progressed in recent years, studies addressing cybersecurity in this area are scarce, being nowadays an open challenge [28]. In this context, there has been a recent attempt to study the problem of cybersecurity in BCI, where there are works that have partially studied specific aspects of cybersecurity in BCI, such as the possibility of disrupting neuronal signaling during neurostimulation [4]. One of these studies [29] has proposed the classification of attacks depending on the field of application of BCI, as neural applications, user authentication [30], entertainment, and video games, and smartphone applications.

A work performed by Landau et al. [31] studied the feasibility of obtaining information about a subject's personality while playing video games using a BCI. This experiment was developed using different *machine learning* algorithms to classify the data captured during the game. Once the data were available, they were compared with those obtained when the subject was resting. With this, they obtained 73% of accuracy, enough to demonstrate that they could violate the privacy of the subjects who had undergone the experiment.

Meng et al. [32] created an experiment, where they focused on the integrity of the captured data, applying deliberate modifications to them. In the same way, Sundararajan [33] developed a laboratory scenario, where the author ran tests with different attacks to the proposed scenario. These attacks were as follows: (1) passive eavesdropping, intercepting the data without the user being aware, (2) active interception, able to collect the data and discard or resend them, (3) denial of service, and (4) data collection, modification, and retransmission to obtain a different response.

Focusing on possible attacks through visual stimuli [34], Martinovic et al. [13] showed four different types of images in their experiment: (1) automated teller machines (ATMs), (2) debit cards, (3) geographical points, and (4) famous people. With these images, the authors sought to obtain private information about the user, especially the user's residence, using the geographic points. The images appeared randomly throughout the experiment, and each image had a duration of 250 ms. Before starting the experiments, the subjects had to pass a training phase, where each user's P300 was classified. For this training, random numbers were displayed, and the user was asked to count the number of occurrences of each number, which was used as a calibration.

Frank et al. [15] tested subliminal attacks effectiveness in extracting private information, following the same protocol as for supraliminal stimuli. The procedure consisted of an initial calibration phase of the BCI using a series of random numbers. The protocol consisted of showing a 15-minute video, taken from the film “The Gold Rush” (1925), with images of former President Barack Obama and another unknown person inserted. They concluded that the results were similar to those obtained previously with supraliminal images, being able to extract information from the subjects without them knowing they were being studied.

Table 1 shows a comparison of the parameters used in this work with respect to the literature. Since these parameters could be different depending on the objective of the studies, they have been compared with works that have a similar purpose, which is compromising the integrity of the user's data. The most relevant parameters have been considered, such as when the images are displayed or the task the subject has to perform.

Although there are studies in the literature on subliminal and supraliminal attacks, the scarcity of studies and the different methodologies used do not allow comparison. Because of this, the next section analyzes subliminal stimuli from a psychological point of view to determine if they are biologically possible.

### 2.3. Subliminal Stimuli

Subliminal stimuli are extremely controversial, with researchers disagreeing on whether they affect human behavior or not. The first time these stimuli were used was in 1972 by the market analyst Karremans [35]. In this experiment, he showed on the screen of a cinema the phrase “Drink Coca-Cola”, and according to his results, the sales of Coca-Cola increased by 20%. Years later, he admitted that he had never conducted this experiment. In addition, such stimuli have been studied before, for example, by Freud [36]. He determined that stimuli could have a small influence on factors such as sleep or wakefulness. Lundy and Tyler [37] indicated that there are subliminal effects in audiences exposed to sound or visual messages when the voice volume is lowered, because this change in perception demands greater, sometimes extreme, attention from the listener. As their perceptual capacity is enhanced, they generally pick up what is meaningful, which is what has been previously encoded with this intention.

Another use of this type of stimulus is called priming [38], an effect related to implicit memory, whereby exposure to certain stimuli influences the response to the presented stimuli [39]. This concept is widely used in the educational field, for example, when a teacher asks students to read the topic before the lesson. This first read improves later attention in class due to the priming effect [40]. However, following this methodology, several experiments have proposed this approach to influence users' decisions [39]. Nevertheless, many other experiments deny that this has a real impact on the user [41].

In general, visual stimuli are not well established, and numerous studies claim they are useless. Pratkanis et al. [42] reviewed more than 200 works and concluded that none of them provided reliable evidence that subliminal messages influence behavior. Many of these works did not find the desired effect, while those finding an effect suffered from methodological flaws. In this regard, Moore [43] stated: “there is no empirical evidence for more substantial subliminal effects, such as eliciting specific behaviors or changes in motivation”. There is some evidence of subliminal perception (not persuasion), i.e., minimal processing of information that escapes the conscious mind. An example of this is the so-called cocktail party phenomenon [44]. This situation consists in increasing the attention of a subject after identifying his/her name, even when the attention was focused on different tasks. This indicates that the brain is processing information without being aware of it. However, so far, no studies have demonstrated the effects on motivation and behavior similar to those claimed by advocates of subliminal persuasion.

To emphasize subliminal stimuli ineffectiveness, Pratkanis et al. [42] conducted a study of retail audio tapes containing subliminal messages aimed at improving either self-esteem or memory. Neither self-esteem nor memory improved in any of the subjects. This experiment was repeated two more times, and the results showed that the subliminal stimuli did not have any effect.

## 3. BCI Framework: Generation, Acquisition, Processing, and Visualization of P300

This section describes the design and implementation details of each element defining the proposed BCI framework, which is graphically represented in Figure 2. The first phase is responsible for *EEG acquisition*, which hosts the software in charge of connecting the BCI device to the computer. In the same way, it saves the acquired data for later processing. Once the data is stored in a file, the *EEG processing* procedures must be performed. The purpose of this phase is to facilitate the study of the P300 in the next stage. For this, it is necessary to follow a series of steps, such as filtering, editing (e.g., downsampling to resample the signal), and labeling the data. Such labeling allows marking the points of interest like stimulus appearance, stimulus disappearance, and time of appearance of the P300. Finally, the last step of our proposal is the *Visualization of the P300*. For this, the framework graphically displays the EEG to allow the identification of the P300 potential, the main goal of this work. Each of the processes that integrate the framework and the functions they perform is detailed below.

### 3.1. BCI Headset

One of the fundamental pillars of this work is the BCI headset, which makes it possible to obtain the brain waves of a subject and develop the necessary experiments. Therefore, the choice of the BCI device is of vital importance for the objective pursued.

The equipment used in this work is the OpenBCI UltraCortex Mark IV EEG Headset [45], which is oriented towards the academic sector. This BCI has several advantages, such as the setup speed, as the BCI configuration is straightforward, or its low cost compared to other devices with similar specifications. However, it cannot be used for medical purposes due to the low number of channels and the limited accuracy of its electrodes. Also, the BCI kit adds electrodes that can be attached to the body, which allows performing *ECG* to measure cardiovascular activity or even study muscle activity (*EMG*).

The OpenBCI UltraCortex Mark IV EEG Headset integrates its intelligence in the Cyton biosensing board. In addition, the BCI is connected to the computer via Bluetooth, where the computer uses a USB receiver, enabling the reception of data. The BCI headset follows the international format *10-20 System* and offers 35 placement positions, which can be seen in Figure 3. Although the interface can use up to 16 electrodes simultaneously, this work considers 8 electrodes. In particular, the locations selected are FP1, FP2, C3, C4, P7, and P8. Additionally, we have used O1 and O2, because they correspond to the occipital area of the brain, responsible for reacting against visual stimuli.

Once the BCI is ready, the next step is to configure the presentation of both known and unknown images. For this, the framework implements a Python script that allows displaying images and marks the timestamp at which it has been exposed. In particular, the script saves, in *Unix Timestamp* format, the starting and ending times of the experiment and the exact time of the stimulus appearance. This will be used in subsequent processes for the labeling of the EEG signal. It is also relevant to mention that the script has several configurations for different experiments, adapting the sample rate of the target images (more details in Section 4). Finally, it is essential to note that, as it is not a static video but a process running on the machine, it may inevitably delay. The idea is to reduce as much as possible the background processes running on the machine and assign real-time priority to the process, both for memory and CPU.

### 3.2. EEG Acquisition

The software used by the framework to acquire the EEG signal is OpenBCI GUI, offered by OpenBCI. This application is the one that best adjusts to our needs, and the simplest one, although it also has some disadvantages. Among the advantages, it allows seeing graphically and in real-time the data received from each electrode, making it easier to perform initial calibration and check that electrodes are touching the scalp correctly. Another advantage is to record the experiments and later reproduce them. These reproductions are possible, thanks to the fact that it saves all the data in a file. Nevertheless, this is also a disadvantage, since the text file format is only understandable by the OpenBCI application, and it is not unique between different versions of the application.

The OpenBCI application offers compatibility with *Lab Streaming Layer* (LSL) communication functionality. LSL [46] is a library designed to allow the transmission of data between different devices. Several tools have been built on top of this library, such as data recording, file import, and applications that allow data from various acquisition hardware (a BCI, for example) to be available on the laboratory network. OpenBCI GUI uses this protocol as a gateway to other applications. In particular, the possibility of reproducing a specific experiment already developed, and its complete transmission via LSL to other software generates a considerable potential for experimentation.

After the reception of the data, the next step is to store all the data into a portable file, which external applications can understand. The file format selected for this purpose is *CSV*. Therefore, an external application is needed to receive the data via LSL and convert it into a CSV file. This functionality is provided by *OpenViBE*, a platform dedicated to the design, test, and use of BCI. OpenViBE is extremely intuitive, since it is based on the so-called “boxes.” Each box offers a specific functionality, such as file writing, data filtering, or graphical representation of the data. This offers the possibility of deploying a complete scenario, which receives the data, processes them by applying the selected filters, and exports them to a CSV file. The proposed solution uses OpenViBE, which assembles a scenario that receives the data through LSL, exporting them to a CSV file.

### 3.3. EEG Processing

The EEG processing phase intervenes after storing the recorded EEG. Our framework uses *MatLab* for EEG processing since it is one of the most widely used software devices for this purpose. There are a large number of plugins that extend the Matlab functionality, with *Letswave* [47] being one of the most used and well known for BCI. Letswave is specially optimized for EEG data and provides multiple functions for processing neurophysiological signals, including data processing and analysis of time- and frequency-domain signals, also presenting a GUI to ease the process. Additionally, it allows the comparison of the data between each of the steps performed, such as filtered and unfiltered data.

After configuring Letswave, the framework imports the data previously stored in the CSV file. Letswave version 7 offers the possibility of importing data from Matlab. Once the data are loaded into the framework, it applies the notch filter at 50 Hz and a band-pass filter between the frequencies of 5 Hz and 30 Hz. Finally, a 5 Hz downsampling is performed, leaving the signal with 50 samples per second (originally 250). *At this point, algorithms for feature extraction such as ICA* [48] *or Bilinear Analysis* [49] *could be applied.*

After processing, the next step is to label the data. For this, one more column is added to the data called “control column” (Figure 4). This column has all values set to zero, except when a stimulus is displayed, which will have a higher value than the rest of the data. In this way, it is easier to discriminate the points of interest in the graphs.

### 3.4. P300 Display

With the EEG data ready for study, the last process of the framework is to plot the EEG and detect possible P300. Several tools are available for this purpose. *Letswave 7* offers a module with a series of functionalities for creating figures and the graphic representation of the EEG. The graphing data module of this tool helps make the first contact and check that the data is correct. However, the generation of figures exported for external use is complex, so this option has been discarded. Thus, the figures have been created with Excel, as it is simpler and meets the requirements for the purposes we are pursuing.

For the visual identification of the P300 potentials, the literature has visually studied the behavior of the signal in terms of voltage and amplitude. The shape of a P300 potential starts with a decrease of the signal, which can reach negative voltage values and then increase the voltage until a peak that will have a slight decrease in the voltage. After this, the maximum voltage peak occurs, in our particular case, usually up to 40 *µ*V.

## 4. Experiments

This section details the design and setup of the experiments performed and the protocol used to conduct them. In this sense, this section offers information about the subjects intervening in the experiments, including relevant personal and medical information. Finally, we compare the results obtained and analyze whether there are similarities between them.

Figure 5 presents the scenario used to validate the framework, whose functionality has been tested with ten subjects. In particular, both target and nontarget images were presented to the subjects wearing a BCI Headset. The cerebral activity captured due to these stimuli was used as input to the implemented BCI framework. Moreover, the personal information of these subjects can be found in Table 2. In general, most of the subjects participating in the experiments had an average of 23.7 years old, being mainly men. Most subjects had no diagnosed neurological diseases, except for one subject who presented hyperactivity and attention deficit disorder.

Five individual experiments were performed on each subject, based on sampling target images differentiated from a more extensive set of nontarget images, with about an 8% probability of occurrence. These experiments aimed to detect whether these target images produced a P300 potential in the subject. The target images have been displayed at the same size as the nontarget images. Likewise, no attempt has been made to hide them, but they have been displayed full screen. The videos shown in the five experiments were a series of images with a total average duration of 50 seconds (depending on the sample time of the target image). The experiments differed on the sampling time of target and nontarget images, decreasing the target images sampling time in each successive experiment (500 ms, 250 ms, 100 ms, 50 ms, and 10 ms). The sample times of the nontarget images remained at 500 ms regardless of the experiment.

The target images were personalities known by the subjects (Figure 6(a)), shown to them before starting the experiment to ensure that they were recognized. Unfamiliar images were neutral images, which the subjects were not familiar with, usually of natural landscapes (Figure 6(b)). These images varied from experiment to experiment, thus preventing them from being recognized by the subjects. Similarly, the number of times the target image appeared was randomized. This is because of what has been studied in state of the art, where it is confirmed that the time between target images influences the generation of the P300.

Concerning the protocol followed for the execution of the experiments, we begin by detailing the environment, in which the subjects were at the time of the experiment. In this sense, a room with as little noise as possible was selected to avoid the subject receiving external stimuli that could generate noise in the EEG or alter the generation of the P300. Subjects were asked to try to avoid all possible movements, especially facial movements. These movements add a significant amount of noise to the data acquired and may cause a P300 wave to be lost. Similarly, they were asked to count the number of occurrences of the target image mentally. This is not necessary to generate a P300, although we ensure that the subject is concentrating on the experiment. Between each experiment, approximately 30 seconds was allowed for the subject to settle back in and check that all electrodes were still in contact with the scalp. It also allowed the subject to pay more attention to the new experiment, avoiding fatigue.

Once the details of the experiments have been presented, we analyze the results obtained from each experiment. To validate the EEG signals acquired, a figure from the literature is taken as a reference, including both P3a (target) and P3b (nontarget) Figure 7. The results obtained for each subject and experiment are shown in Table 3. In this table, three possible types of responses to a target image are identified. The first consists of the identification of a P300 (**✓**), the second is that no P300 has been detected (**✗**), and, finally, a pattern resembles the P300, but it is not possible to confirm it (**?**). The values for each cell represent a value over the total of three or four tests, depending on the experiment. For experiments 1, 3, 4, and 5, there are three occurrences of the target image, while, for the second experiment, there are four events of the target image. The circumstances are different, so that the subject does not always search for the same number of occurrences, and thus provoke a higher P300.

For the first experiment, in which the images were shown for 500 ms to the subjects, at least one P300 wave was obtained in all subjects, indicating that the subjects' brain commonly recognized this duration of the image. In total, for all subjects, 17 P300 waves have been elicited, exceeding 50% of presented P300.

For experiment 2, the target image sampling time was reduced to 250 ms, and the number of times the target image is displayed was increased. In this case, 16 P300 waves have been detected, representing a 40% of occurrence over the total number of target images presented. This is 10% lower than in experiment 1 and may be due to reducing the target image sampling time. However, many factors can influence this reduction, such as subjects' concentration in performing the task.

Experiments 3 and 4, whose sampling time is 100 ms and 50 ms, respectively, present similar results. For these experiments, 50% of P300 waves have been obtained concerning the displayed stimuli. The results between experiments are quite similar, because the stimulus that the subject receives with these sampling times is quite similar (the image cannot be observed too clearly). However, there is an improvement between these two experiments concerning experiment 2, although the sampling time has been reduced by more than half. We highlight that this situation could be caused by the perception that subjects have over the sampling time, where the transition between target and nontarget images is more clearly appreciated than the target image itself.

Finally, experiment 5 reduces the sampling time to 10 ms, representing the situation in which the images are subliminal. The aim is to study whether this stimulus can be processed by the brain or not. In this experiment, some results have been classified as doubtful. This is motivated by certain variations existing in the EEG during the intervals, where the P300 should appear, between 200 ms and 1000 ms after the stimulus, that could be interpreted as P300 potentials. However, this cannot be confirmed to be the case, because they differ with the usual latency and peak voltage. In the same way, according to the literature, where it is stated that these stimuli do not impact brain activity, it is most likely to be noise from other external factors.

The time required to perform the experiments can be divided into two phases. On the one hand, the time needed to generate the EEG and, on the other hand, the time required to process it and display the P300. For the calculation of the total time, the following aspects have been considered: the preparation of the stage and checking of the correct functioning of the material (ten minutes approximately), each sample of images that lasts about five minutes, and two minutes that are left between each video for rest to avoid visual fatigue. This would make a total of 35 minutes for the conduction of all the experiments for each subject. After this, preprocessing is applied, which takes about 20 minutes, while image generation takes 20 minutes per experiment, 100 in total for the five experiments. In summary, for each subject, the total amount of time, starting from the moment when the EEG is captured until it is processed and converted into images, can be calculated as follows: preparation time + (image sampling time *∗* 5 + rest time *∗* 5) + preprocessing time + (image creation time *∗* 5) = 10 + (5 *∗* 5 + 2 *∗* 5) + 20 + (20 *∗* 5) = 165 minutes/per subject.

Analyzing the results in terms of the subjects, and not focusing on each individual experiment, we have observed that older subjects have a slightly longer latency to onset of P300. This may be why there is a reasonably uniform distribution, since the ages are not too far apart (16–31 years). On the other hand, the gender difference does not seem to have affected the P300 potential. However, it is not possible to delve too deeply into the gender difference due to the imbalance between males and females in the experiments.

## 5. Conclusions

This work presents a study of the feasibility of visual attacks aiming to compromise the privacy of the user's data employing the P300 potential. For this purpose, a scenario based on EEG-based BCI technologies has been designed. Therefore, as a contribution of this work, a BCI framework has been developed to supply all the BCI cycle phases. The experiments performed first display known (target) and unknown (nontarget) images to the subject. Simultaneously, the BCI framework receives and stores the EEG sent by the BCI device. Once the data have been stored, they are correctly processed and displayed to detect the existence of a P300 event visually. To test its functionality, five experiments have been designed, tested on ten subjects. In each of these experiments, the sampling time of the target image has been reduced (500 ms, 250 ms, 100 ms, 50 ms, and 10 ms), starting from supraliminal stimuli to subliminal stimuli. It is worthy to mention that a comprehensive and exhaustive configuration of experiments has been performed, improving an important gap existing in the literature and helping understand if subliminal stimuli can generate P300 waves, or not. After the experiments, we have observed that supraliminal stimuli produced P300 over 50% of the time in the subjects. On the other hand, no evidence has been found that subliminal stimuli produce any impact on the users' brains. Some different conclusions have been obtained; for example, a more significant number of P300 were obtained in people with younger age and with a shorter latency.

As future work, we will focus on subliminal stimuli differently, such as hiding them in the video, e.g., following the approach of Frank et al. [15]. On the other hand, we plan to improve the conditions in which the experiments have been performed, using an environment more isolated from external stimuli. Regarding the BCI used, we also plan to increase the number of electrodes used to 16 and use muscle electrodes. In the same way, it is planned to increase the number of subjects participating in the experiment, trying to provide a greater variety between ages or diagnosed diseases. In this way, it will be possible to conclude more clearly whether these parameters affect the P300 potential.

## Figures and Tables

**Figure 1:** Examples of use of P300 evoked potential.

**Figure 2:** Conceptual diagram of the implemented BCI framework.

**Figure 3:** 10–20 system.

**Figure 4:** Adding the control channel to a graph. (a) Graphic without control channel. (b) Graphic with control channel.

**Figure 5:** Scenario deployed for conducting the experiments.

**Figure 6:** Example of (a) target image and (b) nontarget image.

**Figure 7:** Shape of a P300 wave, comparing target and nontarget stimuli.

**Table 1:** Comparison of the parameters used between the literature and this work.

Reference	Number of channels	Stimuli duration	Percentage of target images	Number of images presented	Number of subjects	Task performed
Martinovic et al. [13]	14	250 ms	1	11	30	Visualize images
Frank et al. [15]	8	13.3 ms	2	900	29	Watch a video
This work	8	500 ms, 250 ms, 100 ms, 50 ms, 10 ms	8	60	10	Visualize images

**Table 2:** Information concerning the participants in the experiments.

Subjects	Gender	Age	Mental conditions
Subject 1	M	23	No
Subject 2	M	23	No
Subject 3	M	27	No
Subject 4	M	16	Hyperactivity and attention deficit disorder
Subject 5	M	31	No
Subject 6	M	32	No
Subject 7	M	22	No
Subject 8	M	22	No
Subject 9	F	20	No
Subject 10	F	21	No

**Table 3:** Results of the five experiments performed over ten subjects.

Experiments	Experiment 1			Experiment 2			Experiment 3			Experiment 4			Experiment 5			Summary
	✓	✗	?	✓	✗	?	✓	✗	?	✓	✗	?	✓	✗	?	
Subject 1	2	1	0	3	1	0	1	2	0	1	2	0	0	2	1	7
Subject 2	3	0	0	2	2	0	2	1	0	1	2	0	0	3	0	8
Subject 3	2	1	0	3	1	0	1	2	0	1	2	0	0	3	0	7
Subject 4	2	1	0	1	3	0	1	2	0	3	0	0	0	3	0	6
Subject 5	1	2	0	2	2	0	2	1	0	2	1	0	0	2	1	7
Subject 6	1	2	0	1	3	0	2	1	0	0	3	0	0	3	0	7
Subject 7	2	1	0	1	3	0	0	3	0	2	1	0	0	3	0	8
Subject 8	1	2	0	0	3	0	1	2	0	1	2	0	0	2	1	3
Subject 9	1	2	0	1	2	0	2	1	0	3	1	0	0	2	1	7
Subject 10	2	1	0	3	1	0	2	1	0	1	2	0	0	3	0	8
Summary	17			16			14			16			0			68

Experiments, where a P300 was clearly detected, are marked with a ✓ symbol, whereas those experiments without its detection are indicated with an ✗ mark. Finally, those results that did not clearly present a P300 are highlighted with a “?” symbol.

## Data Availability

The data used to support the findings of this study are available from the corresponding author upon request.
